The article "Observation of Wound Healing Effect and Aesthetic Satisfaction of Patient with Second Degree Burn Wounds Treated by Kangfuxin Solution" was published in 2022. Journal: Evid Based Complement Alternat Med.

# Observation of Wound Healing Effect and Aesthetic Satisfaction of Patient with Second Degree Burn Wounds Treated by Kangfuxin Solution

**DOI:** 10.1155/2022/1664225

**Published:** 2022-07-07

**Authors:** Changhai Liu, Yuren Zhong, Cuie Wei, Fanjun Meng, Yongdong Pei, Xiangsheng Ding

**Affiliations:** Department of Burn and Plastic Surgery, The First People's Hospital of Lianyungang, The Affiliated Lianyungang Hospital of Xuzhou Medical University, Lianyungang 222000, Jiangsu, China

## Abstract

**Objective:**

To study the effect of wound healing and aesthetic satisfaction of patient with second degree burn wounds treated by Kangfuxin solution.

**Methods:**

84 cases of burn plastic surgery in our hospital from October 2020 to October 2021 were included. All patients were randomly divided into observation group and control group with 42 cases in each group. Patients in both groups received basic treatment after admission, and patients in the control group received conventional treatment. Patients in the observation group were treated with Kangfuxin solution after admission. The clinical efficacy, wound healing time, secretion disappearance time, infection rate, and scar formation rate after treatment were compared between the two groups. The scores of patients and observer scar assessment scale (POSAS) before and after treatment were compared between the two groups, and the occurrence of adverse reactions during treatment was also compared between the two groups.

**Results:**

The total effective rate of the observation group was 92.86%, which was significantly higher than that of the control group (61.90%) (*P* < 0.05).The time of wound healing and secretion disappearance in the observation group was significantly shorter than that in the control group (*P* < 0.05); the infection rate and scar formation rate in the observation group were significantly lower than those in the control group (*P* < 0.05).The scores of PSAs and OSAS in the observation group were significantly lower than those before treatment and after treatment in the control group (*P* < 0.05). There was no significant difference in the total incidence of adverse reactions between the observation group (7.14%) and the control group (9.52%) (*P* > 0.05).

**Conclusion:**

The Kangfuxin solution has the advantages of fast wound healing, high patient satisfaction, better therapeutic effect, and high safety, which is worth clinical application.

## 1. Introduction

Burns are caused by various reasons, such as fire, electricity, and chemicals. Various injuries induce the damage of skin and mucosa, which affect the defense function of the skin, causing damage to the body's tissues and organs. Burns are a common injury in everyday life and work [1,2]. Burned tissue may become necrotic. In tissue burns, fluid leaks from the blood vessels causing tissue edema. In large burns, abnormal vascular permeability, loss of large amounts of fluid, and possible shock occur. Effective treatment for the patients with burns admitted to the hospital in time will avoid the adverse consequences. If the treatment is not timely or improper, severe consequences would occur, for instance infection. Severe burns can even lead to the death of the patient.

The article "Observation of Wound Healing Effect and Aesthetic Satisfaction of Patient with Second Degree Burn Wounds Treated by Kangfuxin Solution" was published in 2022. Journal: Evid Based Complement Alternat Med.

Therefore, what are the effective ways to promote the healing of patient wounds and to improve the patient's prognosis have become a key topic of physicians in burn department. The Kangfuxin solution is an ethanol extract of the dried insect body of the American cockroach, which is widely internally and externally used for anti-inflammatory and regulatory immunity. Kangfuxin liquid is a light brown liquid with a slightly fishy smell and a sweet taste. The main component is the extract of dried American cockroaches, which contains various polyols, epidermal growth factor, amino acids, mucoglycosine, and other amino acids and other activities. Substances have the functions of anti-inflammatory, reducing swelling, promoting cell proliferation and growth of new granulation tissue, accelerating the repair of damaged parts, accelerating the shedding of necrotic tissue, and improving the body's immunity. Generally, there are two ways to use the new rehabilitation solution: internal use and external use. Oral administration is mainly for the treatment of digestive system ulcer-related diseases, such as gastric ulcer and duodenal ulcer, as well as the adjuvant treatment of pulmonary tuberculosis and hemoptysis. External application is mainly used for adjuvant treatment of wounds, with anti-inflammatory, detumescence, promoting cell proliferation and growth of new granulation tissue, accelerating the repair of damaged tissue, accelerating the shedding of necrotic tissue, and improving the immune function of the body [3,4]. Therefore, We studied the effect of Kangfuxin solution in the treatment of burn wound, and the satisfactory effect was obtained.

## 2. Materials and Methods

### 2.1. Basic Data

A total of 84 burn patients admitted to the Department of Burn and Plastic Surgery in our hospital from October 2020 to October 2021 were selected and included in the study. All patients were divided into an observation group and a control group by random number table method, with 42 cases in each group. Among the observation groups, there were 22 males and 20 females, aged 32 to 56 years old, with an average of (44.72 ± 10.64) years old; burn sites: 15 cases of face, 23 cases of limbs, and 4 cases of others; cause of burns: 15 cases of hot liquid scald, 12 cases of hot metal scald, and 15 cases of flame burns; control group: 21 males and 21 females, aged 32–56 years, mean (44.50 ± 10.42) years old; burn sites: 16 cases of face, 21 cases of limbs, and 5 other cases; reasons for burns: 16 cases of hydrothermal scald, 10 cases of hot metal scald, and 16 cases of flame burn; There was no significant difference in basic data between the two groups (*P* > 0.05), which was comparable.

The article "Observation of Wound Healing Effect and Aesthetic Satisfaction of Patient with Second Degree Burn Wounds Treated by Kangfuxin Solution" was published in 2022. Journal: Evid Based Complement Alternat Med.

### 2.2. Inclusion and Exclusion Criteria

#### 2.2.1. Inclusion Criteria

① All patients were diagnosed with three degrees of four-degree standards, and they were shallowed by skin II; ② they were 18 to 65 years old; ③ patients and family understood this research purpose and the method, agreed to participate, and signed an informed consent.

#### 2.2.2. Exclusion Criteria

① Allergic to the study drug; ② immunization and blood disease exist; ③ accompanied by severe cardiovascular disease or malignant tumors; ④ burn until admission time >24 h.

### 2.3. Methods

① Basic treatment: after admission, both groups received anti-infection, wound treatment, supplemented blood volume, and corrected acid-base and water-electrolyte imbalance. ② The patients in the control group were given routine treatment after admission: gauze was soaked with iodophor (code number approved by SFDA : H65020365, batch number: 20030531, production unit: Urumqi Iodophor Disinfectant Co., Ltd.) and then applied to the wound surface, covered with oil gauze and then bandaged, dressing changed once a day, and reexamination was performed every 2 days during the treatment period, until the patient's wound healed. ③ After admission, the patients in the observation group were treated with Kangfuxin solution: the gauze was soaked with Kangfuxin solution (Z51021834, production batch number: 20150408, production unit: Sichuan Good Doctor Panxi Pharmaceutical Co., Ltd.) and then applied to the wound. Oil gauze was covered with bandages, and the dressing change time, reexamination time, and medication time were the same as those of the control group.

### 2.4. Observation Indicators

① Comparing the clinical efficacy of the two groups, the two groups were evaluated at 7 days after treatment, and the clinical efficacy was markedly effective: the burn wound was completely healed, with no scar hyperplasia and no infection; scar hyperplasia was without infection; ineffective: no healing of the burn wound, and even infection. ② The wound healing time, secretion disappearance time, infection rate, and scar formation rate were compared between the two groups after treatment, and the wound healing time, time of secretion disappearing, infection rate, and scar formation rate were counted during the treatment period of the two groups of patients, respectively. ③ The patient and observer scar assessment scale (POSAS) [5] scores were compared between the two groups before and after treatment, and the two groups were evaluated at admission and 1 month after treatment, respectively. POSAS scores included patient evaluations scale (patient scar assessment scale, PSAS) and observer scar assessment scale (OSAS), PSAS is evaluated from 6 directions of scar pain, itching, color, thickness, flexibility, regularity, score ranges from 6 to 60 points, the higher the score, the more severe the scar. OSAS evaluates from 5 directions of pigmentation, color, thickness, concavity and convexity, and softness. The score ranges from 5 to 50 points. Evaluation was performed by 5 professional physicians. The higher score indicates the worse scar appearance. ④ Comparing the occurrence of adverse reactions in the two groups during treatment, and counting the incidence of adverse reactions in the two groups during treatment.

The article "Observation of Wound Healing Effect and Aesthetic Satisfaction of Patient with Second Degree Burn Wounds Treated by Kangfuxin Solution" was published in 2022. Journal: Evid Based Complement Alternat Med.

### 2.5. Statistical Method

SPSS19.0 statistical software was used to process the data, measurement data were expressed as ($\bar{x}$ ± *s*), and *t*-test was used for comparison between groups; count data were expressed as (%), and *X*^2^ test was used for comparison between groups, and *P* < 0.05 was considered a statistically significant difference.

## 3. Results

### 3.1. Comparison of Clinical Efficacy between the Two Groups

After treatment, the total effective rate of clinical efficacy in the observation group was 92.86%, which was significantly higher than that in the control group (61.90%), and the difference was statistically significant (*P* < 0.05), as shown in Table 1.

### 3.2. Comparison of Relevant Clinical Indicators between the Two Groups after Treatment

After treatment, the wound healing time and the disappearance time of secretions in the observation group were significantly shorter than those in the control group, and the difference was statistically significant (*P* < 0.05); the infection rate and scar formation rate in the observation group after treatment were significantly lower than those in the control group, and the difference was statistically significant (*P* < 0.05), as shown in Table 2.

### 3.3. Comparison of POSAS Scores between the Two Groups before and after Treatment

The PSAS and OSAS scores of the two groups after treatment were significantly lower than those before treatment (*P* < 0.05). The PSAS and OSAS scores of the observation group after treatment were significantly lower than those of the control group after treatment, and the differences were statistically significant (*P* < 0.05), as shown in Table 3.

The article "Observation of Wound Healing Effect and Aesthetic Satisfaction of Patient with Second Degree Burn Wounds Treated by Kangfuxin Solution" was published in 2022. Journal: Evid Based Complement Alternat Med.

### 3.4. Comparison of Adverse Reactions between the Two Groups during Treatment

There was no significant difference in the total incidence of adverse reactions in the observation group (7.14%) and the control group (9.52%) during treatment (*P* < 0.05), as shown in Table 4. The adverse reactions of the two groups of patients disappeared with the extension of time and the corresponding nursing care.

## 4. Discussion

There are many reasons for the formation of burns. Different patients have different burn areas, locations, and burn degrees. At the same time, affected by factors such as age and personal constitution, the clinical symptoms of patients are also different. In the past treatment, anti-infection, semiexposure, and other methods were mostly chosen to make it heal naturally. However, the new skin formed after natural healing after injury is thin and inflexible, and it is very easy to tear and fall off, causing the patient to repeat the disease and easy to appear. Bacterial infection and scarring not only affect the clinical treatment effect but also affect the aesthetics of the skin [6, 7]. The main purpose of clinical treatment of burns is to promote wound healing, prevent infection and scar hyperplasia, and restore the normal function of the wound. In this study, Kangfuxin solution was applied externally to the wound in the treatment of burn wounds, and its clinical treatment effect and the aesthetics of wound recovery were observed to provide help for the treatment of burn wounds.

The results of this study showed that the total effective rate of clinical efficacy in the observation group after treatment was 92.86%, which was significantly higher than that in the control group, which was 61.90%, indicating that the use of Kangfuxin solution to treat burn wounds could achieve better therapeutic effects. Iodophor is one of the commonly used drugs for clinical treatment of burn wounds. It has antitoxic effect and can be used for disinfection of skin and mucous membranes. Many scholars have reported [8,9]. Kangfuxin solution is composed of a variety of amino acids, polyols, peptides and other ingredients. It has the effect of inhibiting protein and RNA synthesis and can play an anti-infective effect. At the same time, Kangfuxin solution also has the effect of improving blood circulation and promoting granulation growth. The author analyzed the specific mechanism of Kangfuxin solution in the treatment of burn wounds as follows: Kangfuxin solution can chemotaxis into fibroblast aggregation when cells proliferate, promoting the growth of granulation tissue and the formation of new blood vessels [10]; in the process of repair and reconstruction, Kangfuxin solution can strengthen the healing of wounds and promote the recovery of skin structure and function. At the same time, Kangfuxin solution also has the effect of regulating immunity, which can enhance the phagocytic ability of phagocytes and the hemolysin activity of lymphocytes. The physiological balance of the body is of great significance and is beneficial to the healing of burn wounds [11]. In this study, the higher total effective rate of the observation group may be due to the fact that Kangfuxin solution promotes the growth of granulation and regulates the body's immunity while anti-inflammatory, which improves the clinical therapeutic effect. Zhang. et al. pointed out Kangfuxin solution has anti-inflammatory, immune-regulating, and granulation-tissue-promoting effects and is fast and effective in the treatment of in vitro wounds, which is consistent with the results of this study [12].

The article "Observation of Wound Healing Effect and Aesthetic Satisfaction of Patient with Second Degree Burn Wounds Treated by Kangfuxin Solution" was published in 2022. Journal: Evid Based Complement Alternat Med.

The wound healing time and the disappearance time of secretions in the observation group after treatment were significantly shorter than those in the control group, and the infection rate and scar formation rate in the observation group after treatment were significantly lower than those in the control group, suggesting that the use of Kangfuxin solution to treat burn wounds can reduce the incidence of infection and scarring. Kangfuxin solution can be taken orally and externally and play an anti-inflammatory role and promote granulation growth effect and can also affect various cytokines such as growth factors, fibroblasts, trace elements, and epidermal cells and promote wound recovery, thereby shortening wound healing and secretion disappearance time. As for the infection rate and scar formation rate of the observation group after treatment, the author analyzed that it may be that the anti-inflammatory and anti-infective effects of Kangfuxin solution reduce the incidence of infection, while Kangfuxin solution promotes angiogenesis and accelerates the shedding of necrotic tissue. Wang et al. pointed out in an animal experiment that rehabilitation lotion has a significant effect on promoting wound healing and can shorten the healing time of wounds, which is consistent with the results of our study [13].

The PSAS and OSAS scores in the observation group after treatment were significantly lower than those before treatment and after treatment in the control group, indicating that Kangfuxin solution treatment of burn wounds can reduce the incidence of scar formation, the wounds recovered well after treatment, and the patients were highly satisfied. The author believes that this is closely related to Kangfuxin solution accelerating the formation of new blood vessels, promoting the production of granulation tissue, and accelerating the shedding of necrotic tissue, which can effectively reduce the probability of scarring and improve the satisfaction of wound healing. In terms of safety, the total incidence of adverse reactions in the observation group was 7.14% and the control group was 7.14%, and there was no significant difference. It can be seen that the use of Kangfuxin solution to treat burns does not increase adverse reactions and has high safety. This is consistent with the results reported by Heuch and Streak Gomersall [14].

The article "Observation of Wound Healing Effect and Aesthetic Satisfaction of Patient with Second Degree Burn Wounds Treated by Kangfuxin Solution" was published in 2022. Journal: Evid Based Complement Alternat Med.

In summary, the Kangfuxin solution treatment of burn wound is fast, and the infection rate of the treatment is high, the scar formation rate is low, the clinical treatment is improved, and the patient satisfaction after treatment is high, the drug is safe, and it has a high clinical application value.

## Figures and Tables

**Table 1:** Comparison of clinical efficacy between the two groups (*n*, (%)).

Group	Significant effect	Curative	Invalid	Total efficiency
Observation group (*n *=* *42)	22 (52.38)	17 (40.48)	3 (7.14)	39 (92.86)
Control group (*n *=* *42)	18 (42.86)	8 (19.05)	16 (38.10)	26 (61.90)
*X* ^*2*^				11.495
*P*				0.001

**Table 2:** Comparison of related clinical indicators between the two groups after treatment (*n*, ($\bar{x}$ ± *s*)).

Group	Wound healing time (d)	Time of secretion disappearing (d)	Rate of infection (%)	Scarring rate (%)
Observation group (*n* = 42)	8.24 ± 2.43	5.33 ± 1.09	1 (2.38)	2 (4.76)
Control group (*n* = 42)	13.27 ± 4.54	10.70 ± 3.75	9 (21.43)	16 (38.10)
*X* ^*2*^ */t*	6.330	8.912	5.742^*∗*^	13.859
*P*	<0.001	<0.001	<0.001	<0.001

*Note.* ^*∗*^Continuous correction.

**Table 3:** Comparison of POSAS scores between the two groups before and after treatment (points, ($\bar{x}$ ± *s*)).

Group	POSAS			
	PSAS		OSAS	
	After treatment	Before treatment	After treatment	Before treatment
Observation group (*n* = 42)	18.20 ± 5.45	7.44 ± 2.78^①^	15.11 ± 4.13	8.45 ± 2.22^①^
Control group (*n* = 42)	18.24 ± 5.49	10.46 ± 4.21^①^	15.08 ± 4.10	11.27 ± 3.45^①^
*t*	0.034	3.879	0.033	4.455
*P*	0.973	<0.001	0.973	0.000

*Note*. Compared with before treatment, ^①^*P* < 0.05.

**Table 4:** Comparison of adverse reactions between the two groups during treatment (*n*, (%)].

Group	Vomiting	Diarrhea	Bloating	Fever	Headache	Total incidence
Observation group (n = 42)	0 (0.00)	1 (2.38)	1 (2.38)	0 (0.00)	1 (2.38)	3 (7.14)
Control group (n = 42)	1 (2.38)	0 (0.00)	1 (2.38)	1 (2.38)	1 (2.38)	4 (9.52)
*X* ^*2*^ */t*						0.000^*∗*^
*P*						1.000

*Note*. ^*∗*^Continuous correction.

The article "Observation of Wound Healing Effect and Aesthetic Satisfaction of Patient with Second Degree Burn Wounds Treated by Kangfuxin Solution" was published in 2022. Journal: Evid Based Complement Alternat Med.

## Data Availability

The data can be obtained from the corresponding author upon reasonable request.
